# Construction of Glycolytic Regulator Gene Signature to Predict the Prognosis and Tumor Immune Cell Infiltration Levels for Prostate Cancer

**DOI:** 10.1155/2022/9273559

**Published:** 2022-02-22

**Authors:** Ling Zhang, Bin Wang, Zhi-Shun Wang, Yong-Lian Guo, Hao Shen

**Affiliations:** ^1^Department of Pathology, Wuhan No. 1 Hospital, Wuhan, Hubei Province 430022, China; ^2^Department of Urology, Suizhou Central Hospital, Suizhou, Hubei Province 441300, China; ^3^Department of Urology, The Central Hospital of Wuhan, Tongji Medical College, Huazhong University of Science and Technology, Wuhan, Hubei Province 430014, China

## Abstract

Prostate cancer (PCa) is the commonly generated noncutaneous neoplasm among men worldwide. Glycolysis had been validated to promote cancer progression. However, the clinical significance of glycolytic regulators in PCa was not well understood. Here, we discovered that glycolytic regulators were dysregulated in PCa samples using GSE8511, GSE6919, and GEPIA. By detecting the expression of these regulators in PCa samples, we found that SLC2A1, SLC2A3, HK2, PFKFB2, TPI1, PKM2, and LDHA had higher expression in PCa compared with normal tissues. Moreover, both higher expression of TPI1, ALDOA, ENO1, LDHA, and PKM and lower expression of LDHB and HK2 were significantly related to shorter progression-free survival time in PCa. Of note, an 8 gene-based risk score was further constructed and confirmed to have a good performance in predicting progression-free survival (PFS) time in PCa. The signature risk score significantly correlated with NK cell, neutrophil cell, macrophage M2 cell, and myeloid dendritic cell infiltration levels in PCa. After bioinformatics analysis, our data suggested glycolytic regulators participated in the regulation of multiple nonmetabolic biological processes, such as RNA transport, biosynthesis of antibiotics, and cell cycle. We recapitulate that the glycolytic regulator signature was a prospective indicator for prognosis and immune cell infiltration levels in PCa.

## 1. Introduction

Prostate cancer (PCa) was one of the widely occurring malignant neoplasms amid males worldwide [1]. The lethality of PCa ranked fifth among carcinoma-related death in men. Although emerging studies revealed that androgen receptor (AR) signaling functioned crucially in the advance of PCa, the mechanism towards modulating PCa tumorigenesis and development needed further investigation [2]. Previous reports implied that the dysregulation of metabolic could serve as a primary driver in PCa development [3]. Epidemiological investigation showed population with a higher dietary fat intake exhibited a higher PCa morbidity and mortality [4]. It is therefore urgent to uncover prospective metabolic regulators conducing to digging out more new biomarkers for PCa.

As a multifactorial pathema, PCa has the characteristics of abnormal activities of diverse regulatory pathways. Among the pathways, Warburg effect was regarded as one pivotal indicator of cancer cell [5]. Warburg effect indicated that more glucose could be converted into lactic acid by cancer cells other than normal cells even under the supply of aerobic. The dysregulation of glycolytic enzymes consisting of SLC2A1, HK2, PFKFB2, TPI1, ENO1, PKM2, and LDHB had been demonstrated in numerous types of human cancers [6–8]. Meanwhile, a few metabolism regulators comprising MYC, HIF1A, and TP53 were reported to participate in regulating cancer development [9, 10]. For instance, several carcinomas, such as gastric [11], bladder [12], and prostate cancers [13], highly expressed PKM2 (the key glycolytic enzyme). LDHA was upregulated in PCa, and ablating LDHA could result in impediment of PCa progression [14]. Nevertheless, the prognostic value of glycolytic enzymes was not well understood till now.

The immune therapy is becoming the promising method to treat tumors, such as lung cancer, gastric cancer, and colon cancer. Despite the fact that PD-1/L1 has not been confirmed to be efficacious in PCa, several novel immune therapies had been approved. For example, Sipuleucel-T was approved for the treatment of castrate-resistant PCa. Besides this, several other immunotherapies such as ipilimumab and CAR-T cell therapy are in clinical development of PCa. Thus, there was still an urgent need to identify novel biomarkers for immune therapy response prediction in PCa. Immune infiltration had been reported as a crucial factor affecting the efficiency of immune therapy in cancers. In PCa, immune infiltration had been confirmed to influence PCa development. For example, high levels of CD3^+^, CD4^+^, or CD8^+^ cells were found to be protumorigenic. In addition, CD20^+^ B cells were enriched in PCa samples compared to normal tissue. High infiltration levels of IL-23-positive cells correlate with abiraterone effectiveness in PCa. Several factors had been reported to correlate to immune infiltration. For example, GPR30 knockdown reduced macrophage infiltration and M2 polarization in PCa. HCG18 and MCM3AP-AS1 increased abundance of M2 macrophage infiltration in PCa. However, the effect of glycolytic enzymes on immune infiltration in PCa remained to be unclear.

Here, we for the first time validated glycolytic enzyme expression pattern in PCa utilizing public datasets, such as GSE6919, GSE8511, and GEPIA datasets. Then, we determined the expression of glycolytic enzymes in the tissues of PCa. Meanwhile, we also explored the association existing in survival time and gene expression. Finally, we conducted bioinformatics analysis to identify the potential impacts of the dysregulation of glycolytic enzymes on PCa. Collectively, our literature could offer new biomarkers for PCa prognosis.

## 2. Materials and Methods

### 2.1. Public Data Analysis

Normalized GSE6919 and GSE8511 datasets were completely analyzed by robust multiarray average (with RMA) method under R 2.6.2 statistical software with affy package from BioConductor, and then, they were applied to ensure the differently expressed mRNAs [15]. Here, we individually represented and performed the normalization for LCM and homogenized tissue datasets. log_2_-transformed values by RMA indicated normalized gene expression level. A total of 75 metastatic prostate tumor samples, 52 normal samples, and 192 PCa samples were included in the GSE6919 database. A total of 16 benign prostate samples, 13 metastatic prostate tumor samples, and 12 local PCa samples were included in the GSE8511 database. The validation of glycolytic enzyme expression pattern in PCa was performed using the GEPIA database (http://gepia.cancer-pku.cn/).

### 2.2. PPI Network and Module Analysis

PPI information was validated by the STRING database search tool. We defined that the comprehensive score > 0.4 was significant. PPI network construction was completed by Cytoscape software. Plugin molecular complex detection (MCODE) toolset was applied to screen the cytokeratin (PPI) network module according to MCODE scores and node number. *P* < 0.05 meant there was obvious difference.

### 2.3. Tissue Collection

The study was approved by the Research Ethics Committee of the Central Hospital of Wuhan, and verbal consent was obtained from all patients. All samples were collected from the Central Hospital of Wuhan, Tongji Medical College.

### 2.4. RNA Isolation and Real-Time qPCR

qRT-PCR for mRNAs was performed as described previously. The Ct values were normalized using *β*-actin as an internal control. Relative mRNA expression was calculated using the 2− *ΔΔ*Ct method.

### 2.5. Establishment of Prognostic Signature

To establish a prognostic signature, the relationship between glycolytic enzymes and OS was evaluated by LASSO and multivariate Cox regression analyses using glmnet packages in R. The Kaplan–Meier (K-M) survival analysis was performed based on the risk scores. The receiver operating characteristic (ROC) curve was analyzed based on the survival ROC package in R.

### 2.6. Statistical Analysis

All derived data of three independent experiments was represented as the mean ± SD. *T*-test or Mann–Whitney *U* test was utilized to compare the difference existing in different groups. *P* < 0.05 (∗∗) meant there was significant difference with a 95% confidence level. Prism software (GraphPad) was applied to perform statistical analyses.

## 3. Results

### 3.1. Dysregulated Glycolytic Regulators in PCa Patients

As mentioned above, some glycolytic gene expression had been reported to be overexpressed in human cancer samples, but the most glycolytic genes had not been reported in PCa so far. Thus, we applied GSE691930 and GSE8511 two GEO databases to determine whether glycolytic gene levels were differently expressed in PCa tissues, after comparison with those in normal prostate tissues.

GSE8511 database analysis result showed that compared to normal tissues, HK2, PFKFB3, SLC2A1, PGK1, PKM2, and LDHA were upregulated, and PGAM1, SLC2A3, and LDHB were downregulated in PCa (Figure 1(a)). GSE6919 database analysis result indicated that HK2, SLC2A1, PKM2, and SLC2A3 were upregulated, and LDHA, ALDOA, PGAM1, and LDHB were downregulated in PCa (Figure 1(b)). The combined analysis data suggested that HK2, SLC2A1, and PKM2 were increased, while PGAM1 and LDHB were decreased in both datasets.

Next, the GEPIA dataset was applied to validate these analyses based on RNA-sequence data. We observed a similar result that HK2, SLC2A1, LDHA, PFKFB2, TPI1, and ENO1 were upregulated, while PFKFB3, ALDOA, PGAM1, SLC2A3, and LDHB were downregulated in PCa compared to those in normal prostate tissues (Figure 2).

### 3.2. RT-PCR Assay Validation of Glycolytic Regulators' Expression Levels in PCa

RT-PCR assay was then conducted to examine glycolytic regulators' expression levels in 80 normal prostate tissues and 20 PCa tissues. The data indicated that HK2, SLC2A1, PKM2, LDHA, SLC2A3, PFKFB2, and TPI1 levels were higher in the samples of PCa than those in the samples of normal prostate (Figures 3(a), 3(c), 3(e), 3(f), 3(i), 3(k), and 3(l)). In contrast, LDHB was decreased in PCa relative to that in normal prostate samples (Figure 3(j)). However, PFKFB3, ALODA, PGK1, PGAM1, and ENO1 expression was not alternated both in the samples of PCa and normal prostate (Figures 3(b), 3(d), 3(g), 3(h), and 3(m)).

### 3.3. Screening and Verification of Prognosis-Related DEGs

We tried to verify the correlation of the 13 glycolytic regulators with PCa patients' prognosis. We carried out LASSO regression with tenfold cross-validation to obtain the minimum partial likelihood deviance (*λ*_min_ = 0.025)-derived optimal lambda value (Figure 4(a)), which had a relationship to 14 DEGs significantly related to progression-free survival (Figure 4(b)).

We used TCGA dataset to conduct Kaplan–Meier curve analysis for further evaluating the prognostic value of glycolytic regulators in PCa. The glycolytic regulators' median expression was considered as the cutoff to separate PCa into highly expressed and lowly expressed samples.  Figure 4 illustrates that obvious correlation between higher expression of TPI1 (Figure 4(c)), ALDOA (Figure 4(d)), ENO1 (Figure 4(e)), LDHA (Figure 4(g)), and PKM (Figure 4(i)) and longer progression-free survival time was demonstrated in PCa. Meanwhile, our data also revealed that slight association between highly expressed LDHB (Figure 4(f)) and HK2 (Figure 4(h)) in PCa and shorter progression-free survival time was shown in PCa. Our findings implied that the dysregulated glycolytic regulators in PCa were probable promising indicators in prognosing PCa.

### 3.4. Establishing and Estimating the 8-Gene Prognostic Signature

Then, we constructed the 8 gene-based risk score on the basis of their Cox coefficients: risk score = (−0.069)∗EXP (HK2) + (0.1896)∗EXP (PGK1) + (0.1718)∗EXP (PKM) + (0.0105)∗EXP (LDHA) + (0.3124)∗EXP (ALDOA) + (−0.1481)∗EXP (LDHB) + (0.0121)∗EXP (TPI1) + (0.1128)∗EXP (ENO1). Then, we calculated each patient's risk score, and then, we utilized “survminer” R package to acquire the median cutoff point and classified those patients into the high- and low-risk groups (Figure 5(a)). Our data suggested that compared to the low-risk group, the high-risk group showed worse PFS (Figure 5(b)). Furthermore, the area under the curve (AUC) analysis indicated that the 8-gene prognostic signature had well predictive capability in 1-year, 3-year, and 5-year PFS for prostate cancer (Figure 5(c)).

### 3.5. The Glycolysis Signature Could Predict the Tumor Immune Infiltration Levels in PCa

Then, we evaluate the correlation of glycolysis signature risk score with neoplasm immune infiltration levels in PCa. Our results showed higher risk score was significantly negatively related to lower NK cell infiltration levels (Figure 6(a)), neutrophil cell infiltration levels (Figure 6(b)), and macrophage M2 cell infiltration levels (Figure 6(d)) in PCa. However, higher risk score was significantly positively related to higher myeloid dendritic cell infiltration levels (Figure 6(c)) in PCa.

### 3.6. Bioinformatics Analysis of Glycolytic Regulators in PCa

Despite the function of these regulators in modulating glycolysis had been elucidated clearly, the nonmetabolic function of glycolytic regulators in PCa was not yet clear. Herein, we conducted coexpression analysis for glycolytic regulators to identify their downstream targets. Bioinformatics analysis results showed that positively-related glycolytic regulators took part in regulating MAPK cascade, mitochondrial electron transport, NIK/NF-kappaB signaling, cell adhesion, mitochondrial respiratory chain complex I assembly, extracellular matrix organization, Wnt signaling pathway, mitochondrial translational elongation, inflammatory response, and angiogenesis (Figure 7(a)). Glycolytic regulators negatively related were involved in regulating transcription, histone acetylation, cellular response to DNA damage stimulus, covalent chromatin modification, viral process, histone H3-K4 methylation, chromatin remodeling, protein sumoylation, protein polyubiquitination, and DNA repair (Figure 7(b)).

## 4. Discussion

PCa is the commonly generated noncutaneous neoplasm in men worldwide [1]. Despite a few pathways, such as AR signaling [2], Wnt signaling [15], and mTOR signaling [16], identified to be involved in regulating PCa progression, the mechanisms of PCa tumorigenesis were yet elusive. Accordingly, to uncover split-new biomarkers for forecasting PCa still faced the challenge. Here, we focused on evaluating the prognostic value of glycolytic regulators in PCa. We observed glycolytic regulators were dysregulated in PCa samples using GSE8511, GSE6919, and GEPIA. By detecting their expression in clinical PCa samples, we validated SLC2A1, SLC2A3, HK2, PFKFB2, TPI1, PKM2, and LDHA had higher expression in PCa than normal prostate tissues. Interestingly, we found higher expression of SLC2A3 and LDHB in PCa was associated with shorter PFS time in PCa. Bioinformatics analysis indicated that glycolytic regulators took part in the regulation of various nonmetabolic biological processes, such as RNA transport, biosynthesis of antibiotics, and cell cycle.

Emerging studies showed that cancer cells were prone to sustaining energy supply via Warburg effect even under ambient oxygen supply. Multiple enzymes comprising SLC2A1, SLC2A3, HK2, PFKFB2, PFKFB3, ALDOA, TPI1, PGK1, PGAM1, ENO1, PKM2, LDHA, and LDHB were reported to be involved in regulating this biological process. Previous studies reported these glycolytic regulators were dysregulated in multiple types of cancers. For instance, PKM2 was upregulated in cervical cancer [17], and knockdown of PKM2 suppressed cancer epithelial-mesenchymal transition [18]. PFKFB3 was overexpressed in tumor samples and could promote breast cancer xenograft growth [19]. In prostate cancer, a few regulators, such as HK2 and SLC2A3, were indicated to participate in the regulation of PCa progression [20, 21]. For instance, HK2 was involved in the cell growth regulation in PTEN and p53 deficiency-driven PCa [22].

In our context, we discovered HK2, SLC2A1, PKM2, ALDOA, SLC2A1, SLC2A3, HK2, PFKFB2, PFKFB3, ALDOA, TPI1, PGK1, and PGAM1 expression was increased. HK2, PFKFB2, PFKFB3, ALDOA, TPI1, PGK1, and PGAM1 expression was decreased in PCa. Besides, our data suggested that upregulated SLC2A3, LDHB, and PFKFB3 and downregulated SLC2A1 had association with longer PFS in PCa. Moreover, we revealed dysregulation of TPI1, ALDOA, ENO1, LDHA, PKM, LDHB, and HK2 exhibited a correlation with PFS time in PCa. Furthermore, we constructed a new 8-gene glycolytic regulator signature, which could predict the PFS time and tumor immune infiltration levels of PCa. These results showed glycolytic regulators could be thought as newly produced biomarker for PCa prognosis.

Although glycolytic regulators' roles in Warburg effect had been demonstrated clearly, the nonmetabolic function in human cancers needed to be deeply explored. For example, PKM2 promotes ovarian cancer growth though regulating CCND1 and CDKN1A expression [23]. PGK1 could mediate the activation of the AKT/mTOR pathway, thus facilitating lung cancer metastasis [24]. We here firstly explored the nonmetabolic roles of these genes in PCa by coexpression analysis. Our data suggested that glycolytic regulators were involved in regulating MAPK cascade, mitochondrial electron transport, NIK/NF-kappaB signaling, cell adhesion, transcription, histone acetylation, and DNA repair. Oncogenic activation of the MAPK pathway was frequently observed in PCa progression. The recent studies indicated the crosstalk among AR, MAPK, and WNT signaling participated in modulating facilitated PCa growth and drug resistance. Characterization of the genomic landscape of prostate cancer has demonstrated frequent aberrations in DNA repair pathways, identifiable in up to 25% of patients with metastatic disease, which may sensitize to novel therapies, including PARP inhibitors and immunotherapy.

## 5. Conclusions

To sum up, the present study showed glycolytic regulators were dysregulated and associated with the PFS time in PCa. Nonetheless, we still need more validation of these glycolytic regulators' molecular mechanism in PCa, but our study could also provide a new hint of unearthing novel biomarkers for PCa prognosis.

## Figures and Tables

**Figure 1:** Several glycolytic regulators were dysregulated in PCa in two GEO databases. (a) HK2, PFKFB3, SLC2A1, PGK1, PKM2, and LDHA were upregulated, and PGAM1, SLC2A3, and LDHB were downregulated in the GSE8511 database. (b) HK2, SLC2A1, PKM2, and SLC2A3 were upregulated, and LDHA, ALDOA, PGAM1, and LDHB were downregulated in the GSE6919 database.

**Figure 2:** Several glycolytic regulators were dysregulated in PCa in GEPIA databases. (a) HK2, (c) SLC2A1, (f) LDHA, (k) PFKFB2, (l) TPI1, and (m) ENO1 were upregulated, while (b) PFKFB3, (g) ALDOA, (h) PGAM1, (i) SLC2A3, and (j) LDHB were downregulated in GEPIA databases.

**Figure 3:** Several glycolytic regulators were dysregulated in PCa samples. (a) HK2, (c) SLC2A1, (e) PKM2, (f) LDHA, (i) SLC2A3, (k) PFKFB2, and (l) TPI1 levels were higher in the samples of PCa, and (j) LDHB was decreased in PCa.

**Figure 4:** Screening and verification of prognosis-related DEGs. (a) LASSO regression with tenfold cross-validation was used to obtain the minimum partial likelihood deviance (*λ*_min_ = 0.025)-derived optimal lambda value. (b) 14 DEGs were significantly related to progression-free survival of PCa. (c) TPI1, (d) ALDOA, (e) ENO1, (g) LDHA, and (i) PKM were positively related to longer progression-free survival time. (f) LDHB and (h) HK2 were positively related to shorter progression-free survival time.

**Figure 5:** The 8-gene prognostic signature had well predictive capability. (a) The median cutoff of the high- and low-risk groups. (b) The high-risk group was positively related to shorter PFS. (c) The predictive capability of 8-gene prognostic signature in 1-year, 3-year, and 5-year PFS for prostate cancer.

**Figure 6:** The glycolysis signature could predict the tumor immune infiltration levels in PCa. The higher risk score was significantly negatively related to lower (a) NK cell infiltration levels, (b) neutrophil cell infiltration levels, and (d) macrophage M2 cell infiltration levels in PCa. (c) The higher risk score was significantly positively related to higher myeloid dendritic cell infiltration levels.

**Figure 7:** Bioinformatics analysis of glycolytic regulators in PCa. (a) The positively-related glycolytic regulators took part in regulating MAPK cascade, mitochondrial electron transport, NIK/NF-kappaB signaling, cell adhesion, mitochondrial respiratory chain complex I assembly, extracellular matrix organization, Wnt signaling pathway, mitochondrial translational elongation, inflammatory response, and angiogenesis. (b) Glycolytic regulators negatively related were involved in regulating transcription, histone acetylation, cellular response to DNA damage stimulus, covalent chromatin modification, viral process, histone H3-K4 methylation, chromatin remodeling, protein sumoylation, protein polyubiquitination, and DNA repair.

## Data Availability

This study used 5 public datasets, including GSE691930, GSE8511, and GEPIA datasets.
